# Climate Change and Water Crises in Pakistan: Implications on Water Quality and Health Risks

**DOI:** 10.1155/2022/5484561

**Published:** 2022-11-22

**Authors:** Waseem Ishaque, Rida Tanvir, Mudassir Mukhtar

**Affiliations:** ^1^Director Area Study Centre (China), NUML, Islamabad, Pakistan; ^2^Department of International Relations, NUML, Islamabad, Pakistan; ^3^HoD Media and Communication Studies, NUML, Islamabad, Pakistan

## Abstract

Pakistan is vulnerable and most affected by adverse impacts of climate change. The study examines the impact of climate change on Pakistan during the year 2022, resulting into unprecedented heatwave and drought in summers followed by the abnormal rains and floods during monsoon season. Agriculture is the backbone of Pakistan's economy, which has been devastated by both drought and floods. While the flood water is gradually receding, the stagnant contaminated water is causing several health risks for the inhabitants. This research argues that water security is the emerging national security challenge for Pakistan. The article investigates the status of water availability vis-a-vis the burgeoning population, agriculture, and other uses of water. Impact of abnormal melting of glaciers, nonavailability of dams for storage of rainwater, and lack of smart means for agriculture water have been examined to empirically validate the arguments.

## 1. Introduction

Climate change has become international buzzword today and it is “no longer an unfamiliar term, which can be comprehended through personal knowledge, experience, and interactions” [1]. The phenomenon of climate change is largely attributed to human induced actions, more specifically in terms of emissions of greenhouse gases in the atmosphere [2]. Therefore, the phenomena of climate change are producing many threats on the Earth surface, ranging from droughts, heavy precipitation, and heatwaves to unprecedented tropical cyclones [3]. All these disasters have varying degree of impact over different geographical zones, resulting into environmental, health, economic, and social impact. There is no denying the fact that the world we live in today is far more vulnerable and affected by the negative impacts of climate change. However, the greatest health impact is being witnessed in the countries which have least share in greenhouse emissions [4]. There is also strong realization to attend to climate emergency, which is causing water security issues around the globe, and threatens food security, agricultural yield, food supply, and prices with serious implications on sustainable development, poverty, and inequality. The UNICEF warns about the availability and use of water in a nicely crafted statement that “the world needs to get water smart, and everyone has to realize that they have a role to play, and we cannot afford to wait” [5]. The “climate change is happening right now, and its effects are being felt around the world” [6].

Pakistan is vulnerable to the negative consequences of climate change, therefore, susceptible to unusual weather patterns, which can create strategic challenges [7]. The rising temperatures are causing rapid melting of glaciers in northern areas and unusual rains as seen in monsoon this year have created mayhem through floods, unprecedented in Pakistan's history in last 30 years. United Nations Secretary General Antonio Guterres stated that Pakistan is facing “the unrelenting effects of epochal levels of rains and flooding” [8]. The men and material losses are enormous and therefore, Pakistan is likely to face water crisis, food shortages, and serious implications for human security. Reacting to the recent flood situation in Pakistan, the Finance Minister Mr Miftah Ismail stated that “Pakistan is dealing with the worst effects of the climate change, which has caused over US$ 30 billion loss to Pakistan's economy and displacing 33 million people” [9]. This study explores the impacts of climate change on the availability, usage, and storage of water in Pakistan. The drought and floods of year 2022 have been taken as case study for analyzing the impacts of climate change across Pakistan by sampling both rural and urban areas.  Figure 1 shows the sectoral usage of available water in Pakistan.

## 2. Materials and Methods

The year 2022 is unprecedented in Pakistan's history of last three decades. The summers produced extreme temperatures which resulted in unusual melting of glaciers in northern areas of Pakistan resulting in partial collapse of bridge near Hassanabad in Hunza [10] as shown in Figure 2.

Later, the exceptional monsoon rains produced extraordinary floods across the country, with huge men and material losses. The evolving trends indicate that Pakistan is most vulnerable to climate change. The floods have devastated the agriculture, livestock, and infrastructure. The loss to national economy is estimated at US$ 30 billion [11]. The survey and data analyses of past two and half decades reveal that Pakistan confronted from absolute dry and drought situations to devastating floods to the extent of witnessing both phenomenon in one calendar year as happening in the ongoing year 2022. The study has been completed by considering drought and floods data from primary and secondary sources with particular focus on this year. The field visits to rural and urban areas of Sindh, Khyber Pakhtunkhwa (KPK), and Baluchistan were conducted for obtaining the first-hand information and data on the impacts of flood situation. The relevant officials in the ministry of climate change and meteorological offices were also interviewed and their views have been incorporated in the study for developing a comprehensive picture, conducting rationale analyses, and arriving at workable findings. The study is very contemporary and relevant and expected to provide valuable policy guidelines to relevant government ministries in Pakistan as they are grappling with the ongoing flood situation and rehabilitation process.  Figure 3 highlights the vulnerability of Pakistan to climate change risks in the global context, which has been explored further in the study to empirically prove the vulnerabilities and risks.

## 3. Findings

### 3.1. Deciphering the Impact of Climate Change on Pakistan

Climate remains the most debated yet least addressed issue for decades. World leaders have often joined heads to tackle this global phenomenon but with little to no success. From motivational speeches to documentaries and movies on the effects of climate change on the Earth has been narrated time and again but to no avail [13]. The developed countries remain aloof of devastating effects of greenhouse gas emission is causing to the ozone layer. The growing depletion of the ozone layer is resulting in increased Ultraviolet (UV) radiations level on the surface of Earth, which has detrimental impact on human health resulting in cancer and weak immune system [14]. These UV radiations have devastating effect on the agriculture sector as well due to low yield of the crops [15]. Scientists have been talking about the infamous “black hole” in the Antarctic region for years. But the recent research in the year 2022 has discovered a hole in the Tropics (Tropics are the regions of the Earth near the equator) which is seven times bigger than the Antarctic region [16]. The more alarming situation is that, despite all this, the industrialized countries are less concerned by the deteriorating ozone and increase in global warming. Various protocols and initiatives like Kyoto Protocol, Copenhagen accord, and Paris accord had been initiated by the United Nations Framework on Climate Change (UNFCCC). Due to the Sovereign status of the global order, these agreements were not a binding, therefore, the industrial powers contributing the most carbon dioxide and greenhouse gases to the environment withdrew from these accords as it did not serve their economic interests. The major global contributors of the CO_2_ emissions are given in Figure 4:

Figure 4 gives an account for the 10 most polluted countries in the world as of 2020. However, China remains leading in that aspect in the year 2022 as well. United States remain on second number with 4.4 billion tons of CO_2_ emissions, while India is third producing 2.3 billion tons of CO_2_.

According to Figure 5, the above countries might not appear as the top 10 global CO_2_ contributors, but they fall in the top 10 per capita CO_2_ contributors, due to their large-scale reliance on oil and small number of populations. United Nations Secretary General Mr Antonio Gutters paid an official visit to Pakistan on 9-10 September 2002 to show solidarity to flood victims and assess the devastations through field visits and official briefings. He stated that the “nature has attacked Pakistan, which contributes less than 1% of global emissions” [19] while facing the consequences of developed countries emissions and pollution of climate. He further added that “it was outrageous that action to reduce greenhouse gas emissions was being put on the back burner, today it is Pakistan and tomorrow, it could be your country” [20], pointing toward industrialized countries. The Global Climate Index (GCI) 2021 has also vindicated Pakistan's vulnerabilities to climate risks as shown in Table 1 below, where Pakistan stands number 8 [21] in the vulnerability Index. The analysis presented highlights the severe impacts of climate change on Pakistan ranging from extreme heat and drought to dreadful floods. [22].

### 3.2. Examination of Water Calamities in Pakistan

Water is an essential need for ecosystem and human life. In recent times, it has been a growing concern that “precious blue” is becoming inadequate resource for future of human survival [23]. The amount of fresh water has remained constant on Earth surface since last 100 years; however, the access to water resources is unbalanced [24] with the rapid population growth, urbanization, and deforestation. Similarly, other issues, such as technological waste, growing industrialization, global warming, and climate change, all are among the key contributing factors for extreme water scarcity [25]. Although the water scarcity has emerged as a global challenge today, it has severely hit the underdeveloped countries like Pakistan with serious implications on all sectors. Pakistan stands among top 10 severely “high water risk countries” with agriculture as most affected sector [26]. Moreover, roughly 80% of the population is facing grave shortage of water during at least 1 month in a year which is very alarming. Under scarce surface water, ground water resources (last resort to water supply) are being over utilized. If appropriate measures are not initiated in time with “whole of nation” and “whole of government” approach, the situation would get worse in time to come and the entire country will face the severe crises of water scarcity by 2025, by most projections “Pakistan could run dry” [27]. The evolving situation has serious implications on the national security of Pakistan, as it will create challenges for sustainable agriculture production which contributes around 23% of Pakistan's Gross Domestic Product (GDP) and creates job opportunities for around 42% of population [28]. According to the report published by Pakistan Institute of Development Economics (PIDE), Pakistan ranks 14th out of 17 very high-risk countries affected by water scarcity, as more than 1/3rd of available water is wasted due to bad management [29]. Since 1962, after the formalization of Indus Water Treaty (IWT) with India, per inhabitant water availability has plummeted from 5229 cubic meters to about 1187 in 2017, which is continuously on the downward slide [30]. The latest UN report on Pakistan's growing population indicates that by 2050, the population is likely to exceed 366 million [31], which will compound the water demand, which is predicted to reach 274-million-acre feet (MAF) by 2025 against available water supply of 191 MAF. This demand and supply gap would continue to grow year on year basis due to growing population and bad water management [32].  Figure 6 shows graphical representation of expected water situation in Pakistan by 2025 viz-a-viz the population [33].

### 3.3. Analysis on Flood Devastations in Pakistan in Year 2022

Most of Pakistan's economy is dependent on the agricultural sector; however, the industrial sector also contributes a great deal to the economic growth of Pakistan. The growing population is directly impacting the environment as the number of vehicles on roads and the number of industries to accommodate these individuals will also increase. The population of Pakistan at the time of independence was 32.5 million; however, as per the 2021 census, the population has increased to 225 million. Although, Pakistan remains significantly low on the global CO_2_ emissions list, yet the effects of global warming have reached Pakistan in a sweeping manner [34]. The issue that industrialized countries failed to realize that the environment does not belong to a single country and when one country damages the ozone layer, the entire world would pay the price for that. The year 2022 was one such year for Pakistan when the effects of climate change brought heavy rainfalls in Pakistan resulting in major loss of lives, infrastructural damage, and massive economic losses to the tune of US$ 30 billion [35]. The NASA issued satellite imagery on the flood situation in Pakistan, which is given in Figure 7.

Torrential rainfall and flooding have wreaked havoc across Pakistan killing over 1600 people including children and destroying infrastructure. According to statement given by Sherry Rehman Minister for Climate Change: “One third of the country is literally under water, a catastrophe of unknown precedent” The data are given in Table 2 and Figure 8. Therefore, the devastating floods caused by unprecedented impact of climate change have hit Pakistan the most this year seriously impacting all the sectors of economy and society [36].

### 3.4. Analysis on Drinking Water Quality in Pakistan

The quality of available drinking water in Pakistan is in a dreadful state. Both surface and subsurface water sources are contaminated and disease prone [37] in major cities as well as rural areas. In the overall context, per capita the availability of water is decreasing precipitously in Pakistan, and the country is ranked as “water stressed” country and fast heading toward “water scarce” country in coming few years [38]. The evolving situation also creates challenges for availability of water for agricultural production, and daily usage requirements, therefore intensifying the human security issues in Pakistan [39]. Water pollution is the most common word today in Pakistan, which can be ascribed to numerous aspects affecting quality of available water [40]. The common causes are an upsurge in the atmospheric temperatures, with an inbuilt tendency to take heat to the threshold of drinking water, microbes, organic chemicals, nutrients, and heavy metals [41]^.^ The research findings have discovered other factors as well affecting water quality, which include surface debris, sporadic water supply, improper discharge of water supply, proximity of sewage water to drinking water lines, industrial waste which has now become very common in almost all major cities in Pakistan, discharge of untreated sewage water and highly incompetent technical workers and service providers on water disposal projects [42]. The pollution of water due to geological and natural factors depends on the presence of different chemicals and their concentration in the geological formations in selected areas, while anthropogenic pollution is caused by extensive use of herbicides and pesticides, coal mining, oil refining, careless disposal of garbage, and septic tanks [43]. Because of such developments, fresh drinking water is available to hardly 20% of population, while 80% population is content with drinking of contaminated water [44]. The recent floods have further aggravated the situation as vast swaths of land in Pakistan is still under water, which is now contaminated causing several health issues. The ongoing situation has also impurified subsurface drinking water due to seepage of contaminated flood water deep in Earth, and government's inability for effective disposal of sewage water.

### 3.5. Water Security

Food and energy security is directly influenced by water security for agrarian society like Pakistan, which contributes more than 23% in national GDP. Agriculture is the backbone of Pakistan as it employs more than 40 million population and guarantor of breadbasket of the country. Therefore, “the loss of major river systems in the past had a domino effect on the thriving civilizations, which became extinct one after the other” [45]. Pakistan is transitioning from water strained country with declining “per capita fresh drinking water, which is less than 1800 cubic meters per year (m^3^/y) to water scarce country (per capita less than 1000 m^3^/y)” projected by 2035 [46]. Similarly, river water also receding to 800 m^3^/y is expected in 2026 due to growing population. Therefore, “water security is emerging threat for Pakistan” [47]. Pakistan is a lower riparian state reliant on the nature and other countries for river's water. India has constructed more than fifty big and small dams on the rivers coming to Pakistan, which are a constant source of irritation in the bilateral relations and vital for Pakistan's water and energy security. Similarly, Afghanistan is also considering construction of dams on Kabul River, which is likely to create two front dilemmas for Pakistan. The situation is even challenging when viewed in the context of availability of only two major dams in Pakistan, Tarbela, and Mangla which were constructed in late 1960s and 1970s; however, “their capacities are reducing due to silting.” While construction of new dams is highly politicized, charged with massive outrage from political parties and masses, therefore, not likely to happen in near future. It is expected that the availability of less water is likely to increase food shortages and create conflict among the federating units and the federation. Similarly, the negative impacts of climate change can cause melting glaciers and unusual pattern of rains, which may lead to flooding as we are witnessing in year 2022.

### 3.6. Food Security

The Indus Basin, which is the bedrock of agriculture support in Pakistan is seriously threatened by the negative impacts of climate change. The changing weather patterns may result in the reduction of crops yield “(15–20% in cereals) and livestock (20–30%)” [48], impacting negatively the dairy and poultry as the agriculture and livestock sectors are the “backbone of Pakistan's economy, which contributes 23% to GDP and accounts 60% exports of country” [49]. The food security is vulnerable to climate change due to reduction in crops and adversarial influences on livestock. Reduced water in real harvesting season is changing the crops patterns and the lands are vulnerable to droughts and flooding as well, which also create massive migrations. The devastations of ongoing floods have created serious food shortages in Pakistan and inflation is also all time high. Pakistan's Prime Minister has already rung the alarm bells by stating that Pakistan is vulnerable to serious food shortage, and it is feared that essential food items may be imported this year and next year as all cultivable lands are under water [50].

### 3.7. Implications of Climate Change on the National Mosaic of Pakistan

#### 3.7.1. Competition over Water Resources

Agriculture-based economies are heavily dependent on the natural resources of the state. This is extremely critical situation for the state to cope with the needs of the masses and economic challenges when there is a scarcity of sustainable renewable and nonrenewable resources. Countries like Pakistan where socioeconomic challenges, such as rising population, lack of political will, internal security issues, urbanization, lack of public policies for managing population, and natural resources are growing at a faster pace as compared with its economic growth. Even the geographical position of the state near the equator is unable to supplement its growing needs and demands. It is an alarming situation for the Pakistan that in the presence of other socioeconomic challenges, the drastic impacts of climate change have also increased its economic and political challenges, while the insufficiency of water reservoirs is creating serious concerns of inter-provincial disharmony. The rising population has not only affected the quantity of water reservoirs but has also depleted the quality in the same manner. The increase in anthropogenic activities is causing water stress on natural reservoirs, while since independence in 1947, the country is facing persistent decline in the availability of water year on year basis due to multitude of factors examined above. According to the estimates of Mr. Jamshed Iqbal Cheema, Chairman Pakistan Agriculture Scientists Association (PASA), in 1947, the capita water availability was 5600 cubic meters, which decreased by 406% from 5260 cubic meters in 1951 to 1038 cubic meters in 2010 and 877 cubic meters in 2020. The PASA estimates that available water will further deplete by 2025 to a level of 660 cubic meters and by 2050 will reach 575 cubic meters as shown in Figure 9 below [51].

The causes of water shortages in Pakistan exist in two types: (a) incidental causes related to poor water management policies at local level, (b) operational causes include the political conflicts (over the water resources on provincial/institutional level) and the societal differences over water management and distribution. Water issue is not only related with the environmental degradation, but also linked with the social factors as abnormal population growth causes a rise in demand of clean water resources, disturbance of equilibrium between communities, provinces, and water resources distribution. As Pakistan consists of multiple ethnicities and diversified geographical terrain but competition over the access of water resources has often created tensions and conflicts among the federating units. The growing vulnerabilities of communities over the insufficiency of water reservoirs promote lawlessness, antistate sentiments and sense of deprivation among its own nationals. Due to lack of strong monitoring mechanism over channelization of available water, for creating a balanced approach between demand and supply of available water, the population is incentivized for illegal water proliferation. The tacit approval from the water management departments has resulted in water theft cases mostly in Southern Punjab and interior Sindh, as there are many illegal drillings, hidden pipelines, and unrecorded water connections from main supply lines. Such illegal water channels mostly exist adjacent to sanitation systems in cities and rural areas, contaminating the available water. The increase in anthropogenic activities is also causing water stress on natural reservoirs.

Another reason of growing water scarcity is unlawful construction and sanitation systems near or over the water channels, which continuously contaminate water, especially during floods blend these altogether. The role of administration is highly crucial in this matter to control such catastrophic constructions and lessen the pressure on water consumption. The unprotected constructions along rivers, lakes, and streams often cause blockage of natural water channels particularly in monsoon and rainy season resulting into loss of lives, roads network, and infrastructure damage as the enormity of flood damages to clean water channels is immeasurable. In 2010 floods, Pakistan witnessed unimaginable losses as around 20 million people were victims, 1.7 million died, 436 healthcare centers were devastated, 80% food reserves were smashed, 2.9 million households were severely damaged, nearly 1.1 million houses were damaged and $ 9.7 billion economic loss in 135 districts. While the issues of accessing the safe water channels was still in demand after flood (96.8% before vs 96.7%). In year 2022 floods, these losses have increased manifolds and caused unprecedented damages to natural water resources. Around 33 million people are direct victims, death troll rising above 1500, while 110 district of Baluchistan (Quetta, Pishin, Killa Saifullah, Nushki, Jaffarabad, and Washuk), Punjab (Koh *e* Suleman ranges, Rajanpur, D. G Khan), Sindh (Mirpur Khas, Thatta, Sajawal, and Shaheed Benazir Abad) and Khyber Pakhtunkhwa (Swat and lower/upper Dir) are declared as most calamity hit areas. While 30% water channels are severely affected, and 63% flood victims are struggling for sufficient clean water channels. The economic losses suffered have been estimated to the tune of US$ 30 billion. The analyses amply highlight the insufficiency of available water and demand, compounded by adverse effects of floods during this year.

#### 3.7.2. Negative Impact on Agriculture Sector

Pakistan is heavily relying on agricultural sector for its international exports and domestic food demands, but in the presence of water crisis and conventional irrigation system for its agricultural production, the country will face severe challenges of water scarcity in times to come. According to Global Food and Security Index 2021, Pakistan ranked 80 out of 113 countries [53] and Global Food and Security Index 2022, it has further slipped by four numbers and now ranks 84 out of 113 countries [54]. Pakistan lags behind all South Asian countries in food insecurity. The lack of progress in agricultural sector is also linked with the mismanagement of land and water resources, unsatisfactory policies of water governance, exponential population growth, and the negative impacts of climate change. Pakistan has also failed to adopt new strategies like advanced water management in agricultural sector, usage of adaptation methods in yields productions to enhance water consumption in eco-friendly manner, educate farmers about the water recycling and water productivity techniques. While water scarcity is a highly charged political issue in Pakistan as there is a turf war between the provinces and the federation. However, Punjab government took good initiative and introduced national water policy of Pakistan to ensure regularization of water governance system in the country. In the presence of fragile agriculture sector development, climate degradation impacts have worsened the livelihood and yield production. Therefore, on a year-on-year basis, the agriculture yield is squeezing, demand of water is increasing, and unplanned urbanization is resulting into loss of precious agriculture land. The overall impact of these issues is creating negative repercussions on agriculture production and aggravating food security situation in Pakistan.

#### 3.7.3. Water Quality and Public Health Risks

The availability of clean drinking water is biggest national security challenge for Pakistan today. The water proliferation and loss of water supply sources from government record is not only raising the administrative issues but also causing multiple public health problems. The contamination of water along with the presence of sanitary pipelines expose the population with the contagious and chronic diseases like diarrhea, cholera, jaundice, typhoid, hepatitis C, liver cancer, and gastrointestinal infections. The water scarcity in Pakistan has enormous impact on health care system as well as the country is struggling with the diseases that are almost nonexistential in developed countries. The significant findings of this study are that in Pakistan, 50% diseases spread through contaminated water and provide most suitable medium of spread and transfer various bacterial and viral infections from human to human or animals to human as the country is facing the 40% of mortality rate caused by the contaminated water intake, while the frontline victims of waterborne diseases are pregnant women, newly born babies, and early teenage groups. It is also important to note that the primary source of water in Pakistan is sub-surface water channels, which over a period have become the hub of different variants of pathogens. According to World Health Organization (WHO) report, approximately, 2.5 million deaths occur annually in Pakistan from widespread diarrheal diseases caused by bacterial and protozoan agents present in inferior quality of drinking water. Around 80% population is exposed to unsafe water as UNICEF Pakistan has also shared the alarming fact that the well-being and health standards of youngsters are at risk; therefore, each year, 53,000 children under the age of 5 years lose their lives due to unhygienic water as 70% of household work and domestic usage of water in Pakistan is dependent on bacterial water sources. The floods of 2022 have compounded the problems of availability and access to clean drinking water. The field visits to rural and urban Sindh, KPK, and Baluchistan vindicated scarcity and contamination of drinking water, which has been reported by several NGOs and media as well. The stagnant water has been contaminated due to mixing of sewage water and created ideal breading grounds for bacteria causing serious health risks. Nonavailability of compatible medical support, inaccessibility, and nondisposal of flood water have created many health risks and entire population in affected areas is vulnerable to adverse effects of contaminated water. In most areas, the disposal of flood water is left to the nature and the government agencies have demonstrated inability to manage it, therefore, spread of waterborne diseases will continue for prolonged period in future.

## 4. Policy Recommendations

### 4.1. Legislation for Interministerial Coordination

The ministry of climate change should take a lead role and coordinate with all the provinces on the issues of water security. All related agencies and departments should work in harmony with this ministry for synergetic response. Similarly, international engagements would be essential component for successful policy implementation; therefore, Ministry of Foreign Affairs and Ministry of Climate Change should remove overlaps and avoid duplications wherever required.

### 4.2. Proper Enforcement of Legislation

“Pakistan Water Apportionment Accord 1991” highlights the judicious distribution of Indus River System (IRS) water among the federating units of Pakistan. However, this accord was unable to deal with the conflicts arising due to unfair distribution of water at times. To resolve this issue, “Indus River System Authority” (IRSA) was established in 1992 [55], through an act of Parliament to work as an institution for Indus water resources regulation and monitoring in Pakistan. However, the problems related to fair water distribution, monitoring and installation system, and the treatment plants lagged during the implementation phase. There always remained issues between Punjab and Sindh regarding unfair water theft. Despite establishment of “Council of Common Interest” (CCI) to resolve the grievances of provinces, but issues persist due to weak implementation mechanism and weak governance. The devolution of power under 18th amendment of the constitution, devolved the water distribution among the rural and urban areas of each province as an internal matter of the provinces; however, water crises remain at large seriously impacting inter-provincial harmony. The Pakistan Council of Research in Water Resources (PCRWR) is assigned the task of ensuring clean drinking water across Pakistan. Implementation of water-related policies requires a great deal of realization and urgency on the part of the political elites of Pakistan. The gravity of the issue needs to be addressed as a national emergency, otherwise, Pakistan is vulnerable to water scarcity situations normally witnessed in African continent.

### 4.3. Judicious Distribution of Water

Being a lower riparian, Sindh is often complaining about the water shortage, especially in the pre-monsoon period each year. The claims made by Sindh government at numerous occasions regarding Punjab stealing its share of water have been denied by Indus River System Authority (IRSA). After the 18th amendment, the allocation of resources to the provinces has been ensured to be judicious; however, the internal distribution of these resources to the rural and urban areas is the responsibility of the provinces. The IRSA is mandated to address, regulate, and develop standard operating procedures (SOPs) for water allocation to the provinces. Regrettably, each province has its own peculiarities in terms of agricultural needs and population, therefore, making the interpretation and implementation of the accord more difficult. To resolve water distribution issues on sustainable basis, the “whole of government approach” is recommended along with on-site consultative visits by the representatives of provincial and federal governments and political leaders for expeditious resolution of conflicting issues. Creating unnecessary fault lines is detrimental to national integration, which should be avoided at all costs.

### 4.4. Water Treatment Plants and Recycling of Water

Pakistan is in dire need of installing treatment plants as every year, hospitals are flooded with patients, both adults and children suffering from diseases resulting from contaminated water. People living in both urban and rural areas are exposed to contagions and microbial bacteria, which enter the body through water, unsafe for drinking. Not everyone in Pakistan can afford bottled water, therefore, it is the responsibility of the state to provide its citizens with safe drinking water. As we know that Pakistan receives a major portion of heavy rains between the months of July to September, where majority of rainwater ends up in rivers, ponds, while the rest of it results in heavy floods of cities and inhabitants. The government through installation of treatment plants can filter clean drinking water for ensuring public health. Similarly, more wastewater recycling plants are the need of time, which should be installed at priority. In rural areas, wastewater treatment is almost nonexistent, leading to pollution of surface and groundwater [56]. The government should pay instantaneous attention to the evolving challenges of treatment of wastewater for sparing clean water for drinking purposes and balanced delivery of recycled water to other uses like irrigation.

### 4.5. Climate Emergency and Disaster Response Mechanism

Pakistan was successful in convincing the world leaders during recently concluded United Nations General Assembly (UNGA) sessions about vulnerabilities to climate risks and the unprecedented impact during year 2022. UN Secretary General Antoni Guterres and US President Joe Biden personally appealed for help for Pakistan to alleviate the suffering and quick rehabilitation of flood victims. It is suggested that Pakistan should consider climate diplomacy as an urgent priority and initiate the process of engagement at bilateral and multilateral levels with developed countries to reduce the vulnerabilities and risks of climate change. Additionally, the disaster response mechanism also needs to be re-energized with strong interagency coordination. The existing structure of national and provincial disaster management authorities should be reinforced through capacity building and professional training. Appropriate equipment for rescue and relief operations also needs to be provided at vulnerable sites for immediate response to save maximum lives. The infrastructure development in flood affected areas should be expedited for which essential resources should be mobilized well in time. Such preparations should be done and rehearsed every year during pre-monsoon season for synergetic and a befitting response to minimize reaction time and save maximum lives.

## 5. Conclusion

Climate change is the evolving global threat, and Pakistan is most vulnerable from its negative impacts. The year 2022 witnessed extreme drought on one hand, followed by unusual floods over the short span of 2-3 months. Therefore, for Pakistan, alarm bells are ringing to take the holistic stock of situation by declaring climate emergency and adopt “whole of nation” and “whole of government” approaches for a comprehensive response ensuring strong interagency cooperation and capitalizing on the synergetic application of all Elements of National Power (EoNP) for optimum results. It is essential to integrate the respective departments under the umbrella of national and provincial disaster response agencies for harmonious functioning, coordination, and execution. There is dire need to create strong national realization to “conserve, preserve, and proportionally distribute existing water resources” [57]. Moreover, smart means for spending agriculture water and recycling of water for uses other than drinking would be helpful as such practices have been adopted by most of developed countries. The construction of more water reservoirs is the need of time and current floods across Pakistan are the testimony of this fact. It is felt that this study shall help the relevant government ministries as an academic policy input for addressing water security issues in Pakistan on sustainable basis.

## Figures and Tables

**Figure 1:** Sectoral distribution of water consumption in Pakistan.

**Figure 2:** Partial collapse of Hassanabad bridge.

**Figure 3:** Climate risk indexing and Pakistan's vulnerability [12].

**Figure 4:** 10 most polluted countries as of 2020 [17].

**Figure 5:** 10 most polluting countries per capita 2022 [18].

**Figure 6:** Water availability in Pakistan by 2025 taken from Dr Muhammad Ashraf's research report.

**Figure 7:** NASA satellite imagery of floods in Pakistan, September 01, 2022.

**Figure 8:** Flood devastation in Swat (KPK) and Baluchistan.

**Figure 9:** Per capita availability of water reservoirs in Pakistan [52].

**Table 1:** Global climate index 2021 [22].

Cri	Country	Cri score	Fatalities	Fatalities per 100000 inhabitants	Losses in millions US$ PPP	Losses per unit GDP in %	Number of events 2000–2019
2000 2019							
(1999 2018)							
1 (1)	Puerto Rico	7.17	149.85	4.12	4149.98	3.66	24
2 (2)	Myanmar	10.00	7056.45	14.35	1512.11	0.80	57
3 (3)	Haiti	13.67	274.05	2.78	392.54	2.30	80
4 (4)	Philippine	18.17	859.35	0.93	3179.12	0.54	317
5 (14)	Mozambique	25.83	125.40	0.52	303.03	1.33	57
6 (20)	The Bahamas	27.67	5.35	1.56	426.88	3.88	13
7 (7)	Bangladesh	28.33	572.50	0.38	1860.04	0.41	185
8 (5)	Pakistan	29.00	502.45	0.30	3771.91	0.52	173
9 (8)	Thailand	29.83	137.75	0.21	7719.15	0.82	146
10 (9)	Nepal	31.33	217.15	0.82	233.06	0.39	191

**Table 2:** Province wise loss suffered because of heavy rain fall [36].

Province	Death toll	Fully damaged	Injured	Economic loss
Punjab	188	16,590 houses	2023	Agricultural
Baluchistan	253	17,608 houses	164	Agricultural
Sindh	422	307,306 houses	1101	Agricultural
KPK	264	30,233 houses	327	Agricultural

## Data Availability

The data used to support the findings of this study are included within this article.
